This article has been retracted.

# Construction and Implementation of Procedural Nursing System for General Surgery Laparoscopic Surgery Based on Deep Learning

**DOI:** 10.1155/2022/8237620

**Published:** 2022-04-21

**Authors:** Yonghong Zheng, Xufang Cheng, Jingtao Shao

**Affiliations:** ^1^Outpatient Office, Chun'an First People's Hospital, Chun'an 311700, China; ^2^Department of Nursing, Chun'an First People's Hospital, Chun'an 311700, China; ^3^Department of General Surgery, Chun'an First People's Hospital, Chun'an 311700, China

## Abstract

In order to explore the construction and implementation effect of a procedural nursing system for laparoscopic surgery in general surgery based on deep learning, this article selects 150 cases of laparoscopic surgery patients admitted to our hospital from January 2020 to January 2021 for research. According to the time of enrollment, the control set and the study set were included in order, with 75 cases in each set. The control set was given routine nursing methods, and the research set was given the management of programmed nursing system based on deep learning. The nursing quality, pain, postoperative recovery, and incidence of complications were compared between the two sets. Logistic regression multivariate analysis of the risk factors for postoperative complications in patients undergoing laparoscopic surgery in general surgery was performed. Based on deep learning, the construction of the procedural nursing system for laparoscopic surgery in general surgery is applied to the nursing management of general surgery laparoscopic surgery, which can improve the quality of care and the VAS score of the patient's pain level, and reduce the incidence of complications. Underlying diseases and routine nursing are risk factors for complications of general surgery laparoscopic surgery, suggesting that corresponding prevention and control work should be done in the procedural nursing of general surgery laparoscopic surgery based on deep learning.

## 1. Introduction

General surgery is the most common and widely used conventional surgical treatment. With the development of medical technology, laparoscopic surgery has become more and more widely used in general surgery. It has notable advantages, including small wounds, less bleeding, and faster recovery. It is very popular among patients [1]. Although general surgery laparoscopic surgery is minimally invasive, there are still problems such as pain and complications after surgery. How to further highlight the minimally invasive features of laparoscopic surgery, reduce postoperative complications, speed up recovery, and provide a high-quality, high-efficiency, and low-cost medical service model is a topic worthy of research by general surgical nurses [2]. Programmed nursing is a planned, continuous, and comprehensive overall nursing model that provides nursing care to patients in the order of assessment, problem determination, planning, implementation, and evaluation, with the purpose of meeting the physical and mental needs of the nursing object, restoring or enhancing the health of care recipients [3]. The deep learning-based surgical complication evaluation system involves the technical field of medical assistant decision-making. The specific scheme includes a cloud database, a cloud server, a medical detection module, a medical case module, and a physician terminal; the cloud database includes historical clinical data of medical units, but at present, there are few applications of deep learning-based procedural management in surgical laparoscopic surgery nursing [4]. Based on this, this article will build a general surgery laparoscopic surgery procedural nursing system based on deep learning and analyze its application effect. The purpose is to provide a theoretical basis for the application of procedural nursing in general surgery laparoscopic surgery in the future.

## 2. The Proposed Scheme

### 2.1. General Information

This article selected 150 patients who underwent laparoscopic surgery in our hospital from January 2020 to January 2021 for the study. According to the time of enrollment, the control set and the study set were sequentially included, with 75 cases in each set. The control set included 45 males and 30 females, ranging in age from 21 to 68 years, with an average age of (45.62 ± 5.87) years. The surgical types were as follows: 37 cases of biliary surgery, 23 cases of gastrointestinal surgery, 10 cases of groin surgery, and 5 cases of other operations; the research set included 46 males and 29 females, with an age range of 21 to 69 years and an average age of (46.85 ± 5.96) years. Six cases of other operations were performed; the age and type of operation of the two sets of patients were compared, and there was no notable difference between the general data, and all patients signed the informed consent.

Inclusion criteria are given as follows: (1) elective laparoscopic surgery; (2) preoperative examination, no contraindications; (3) no immune or endocrine system diseases; (4) no coagulation dysfunction; normal communication with medical staff; and (6) all patients gave informed consent. Exclusion criteria are given as follows: (1) pregnant or breastfeeding; (2) malignant tumor; (3) heart and kidney disease and other important organ diseases; (4) immune system or hematopoietic dysfunction; (5) mental abnormality and neurological disease history; and (6) incomplete clinical data.

### 2.2. Research Methods

Control set: The patients in this set were given routine care in the past, including equipment and instrument preparation before surgery, perioperative health education, disease observation, and complication prevention.

The research set carried out programmed nursing based on deep learning based on routine nursing. Recommended measures were developed by a deep learning-based procedural nursing system for laparoscopic surgery in general surgery.

(1) Programmatic nursing based on deep learning involves a wide range of medical assistant decision-making technologies, mainly including cloud database, cloud server detection, medical detection module and medical record module, and doctor terminal, among which cloud data mainly includes medical units and history clinical data. The procedural nursing system for general surgery laparoscopic surgery based on deep learning mainly closely links and combines artificial intelligence and medical care, and mainly checks and consults the following contents of patients: common symptoms in the patient's medical record, synonyms for symptoms, and common symptoms. The prediction of physical examination and examination items and surgical complications has the advantages of individualizing the overall management and control and intelligent prevention. The use of deep learning in the procedural nursing of laparoscopic surgery in general surgery can quickly predict and test the type, time, and severity of complications, and can complete the test of a patient's medical record and laboratory data within 8 to 12 seconds. The technical background is responsible for receiving relevant data, formulating relevant nursing content for the patient in combination with the patient's nursing recommendation, and forwarding the report to the attending doctor to avoid postoperative complications.
(2) According to preventive measures (high-level evidence), the following programmatic nursing measures are recommended for patients:
  ① Nursing plan formulation: first, the responsible nurse and the nursing team leader need to integrate the information content collected and detected by the deep learning-based general surgery laparoscopic surgery procedural nursing system, and analyze the patient's comprehensive needs management, and formulate targeted care for patients according to the recommended measures, and then push the preliminary programmed nursing measures to patients, discuss nursing measures with patients and their families, and verify and modify some details to ensure patient procedures, and individualized and targeted care measures.
  ② Programmed nursing implementation measures: (a) preoperative cognitive intervention. First, health education is carried out according to the recommended measures formulated by the deep learning-based general surgery laparoscopic surgery procedural nursing system, and the causes and development of the disease, and the principles and advantages of laparoscopic surgery, are explained and introduced to the patients in detail. The patient will be explained and analyzed according to the complications pointed out based on deep learning, and will further formulate intervention measures through the communication results; explain the operating physician to the patient, including the qualifications of the physician, experience, etc., to encourage patients to actively receive treatment and reduce their negative emotions. (b) pain care: During the nursing process, guide patients to describe their feelings after surgery, give patients an attitude of encouragement and comfort, and enhance their confidence in recovery; they can distract patients' attention through music or chat, so as to relieve patients' pain and suffering. Combined with the actual condition of the patient, the paper suggest inhale oxygen to the patient, improve the patient's blood oxygen saturation, and guide the patient to carry out corresponding exercises to enhance autoimmunity. (c) Diet guidance intervention: after the patient completes the operation and wakes up from anesthesia, the patient needs to be given normal saline 6 hours later; 1 day after the operation, a light liquid diet with an intake of 600–1200 ml; 2 days after the operation, liquid or semiliquid food is given, and the intake is 1200∼2000 ml; the diet plan mainly follows low-fat, sodium, sugar, high-vitamin, carbohydrate, and protein, and the ingested food needs to be digestible. The choice of liquid diet is mainly fruit juice and light soup. Patients should be observed for adverse symptoms, including nausea, vomiting, or bloating, while they are eating. (d) Rehabilitation training: six hours after the operation, the patient's condition is basically stable, and appropriate abdominal massage can be given to the patient. First, help the patient to find a stylist posture, take a supine position, and use a hot water bottle with a temperature of 50∼60°C to avoid scalding the patient. The hot compress is completed. Afterwards, the medical staff needs to massage the patient's upper abdomen clockwise with the palm of their hand. The massage intensity should be mixed and tolerated, but it should be noted that the incision area of the patient should be avoided during the massage. At the same time, patients are encouraged to get out of bed as soon as possible, and they are instructed to exercise their lower limbs. After 2 days, they are instructed to practice standing and sitting. When the patient finishes getting out of bed, the catheter can be removed, but the patient's vital signs need to be monitored during this period. Monitor and instruct the patient to perform the exercise training step by step.

### 2.3. Observation Indicators

1. Nursing quality: the hospital's self-made nursing quality checklist is used, including five aspects: nursing behavior, nursing documents, environmental management, operational skills, and safety management. The score ranges from 0 to 100 points. The higher the score, the better the nursing quality.
2. Pain condition: the visual analogue scale (VAS) [5]was used to evaluate the postoperative incision pain of the patients. The score ranged from 0 to 10, with 0 indicating no pain and 10 indicating severe pain. The pain conditions at different stages of the two sets were compared.
3. Postoperative recovery [6]: the postoperative bowel sounds recovery, anal exhaust, defecation time, and hospitalization time were compared between the two sets.
4. Complications [7]: complications include pulmonary infection, urinary tract infection, incision infection, urinary retention, and intestinal obstruction. Urinary retention: after removing the catheter and urinating 2 to 3 times, the residual urine volume was measured. If it was more than 100 mL, it was recorded as urinary retention.
5. Logistic regression multivariate analysis of the risk factors for postoperative complications in patients undergoing laparoscopic surgery in general surgery [8].
6. The cumulative disease readmission rate after one-year follow-up between the two sets was compared.

In this study, all the data were sorted, and a corresponding database was established for it, and all the databases were entered into SPSS 26.0 for data processing, and the measurement data were tested for normality. Multiset test is *F*, repeated measures is analyzed by MANOVA spherical analysis, between sets is *t*, non-normal is Mann–Whitney *U* test; rate is expressed as%, test is *χ*2, and when *P* < 0.05, the difference between data is considered statistically significant.

## 3. The Experimental Result

### 3.1. Comparison of Two Nursing Quality Scores

After the completion of nursing, there were differences in the scores of nursing quality between the two sets, mainly because the five scores of the research set were notably higher than those of the control set, including nursing operation, psychological support, health guidance, nursing documents, and safety management (all *P* < 0.05) [9, 10].  Table 1 shows the comparison of nursing quality scores.

### 3.2. Comparison of Postoperative Rehabilitation Indicators

After the completion of nursing, there were notable differences in perioperative rehabilitation indicators, mainly as the intraoperative blood loss, anal exhaust time, first defecation time, first self-activity, and hospitalization time in the study set were notably lower than those in the control set (all *P* < 0.05) [11, 12].  Table 2 displays the comparison of perioperative rehabilitation indicators.

### 3.3. Comparison of VAS Scores between the Two Sets of Patients after Surgery

At 2 hours after operation, the VAS scores of the two sets were higher, and the difference was not statistically notable (all *P* < 0.05).  Table 3 displays the comparison of VAS scores at different time points after operation.  Figure 1 shows the comparison of VAS scores at different time points.

### 3.4. Comparison of the Incidence of Postoperative Complications

After operation, the incidence of complications in the control set was 20.00%, which was notably higher than that in the study set (4.00%), and the difference was statistically notable (*P* < 0.05), as shown in Table 4.

### 3.5. Univariate Analysis of Postoperative Complications

There are notable differences in age, operation time, underlying diseases, and complications in nursing methods. The main manifestations are that age >60 years, operation time ≥3 hours, and the incidence of complications in patients with underlying diseases and routine care be notably higher than that in patients aged ≤60 years. The operation time was less than 3 hours, there was no underlying disease, and the patients are with deep learning-based programmed nursing (*P* < 0.05), as shown in Table 5.

### 3.6. Logistic Regression Multivariate Analysis of Risk Factors for Postoperative Complications in Patients with General Surgery Laparoscopic Surgery

The multivariate analysis assignment scale is shown in Table 6. Complications are used as the research dependent variable, and age, operation time, underlying diseases, and nursing methods are used as independent variables, and the model is selected based on the actual clinical situation. The results of the logistic regression model analysis show that age >60 years, operation time >3 hours, underlying diseases, and routine nursing were risk factors for complications of general surgery laparoscopic surgery (*P* < 0.05).  Table 7 shows the logistic regression multivariate analysis of risk factors for postoperative complications in patients undergone general surgery laparoscopic surgery.

### 3.7. Cumulative Readmission Rate within 1 Year after Operation

Both sets of patients were followed up for 12 months, and the deadline for follow-up was December 2021. The cumulative admission rate of the control set was 24.00% (18/75), which was notably higher than the cumulative admission rate of the study set of 4.00% (3/75), and the difference was statistically notable (*P* < 0.05).  Figure 2 displays the cumulative readmission rate within 1 year after surgery.

## 4. Experimental Result Analysis

In the process of clinical general surgery, laparoscopic technique is relatively common. This operation belongs to a minimally invasive surgical treatment. Compared with the previous conventional laparotomy, laparoscopic surgery has strong advantages, including smaller postoperative wounds and faster recovery, and short hospital stay and other advantages make this operation recognized by the majority of medical staff and patients. However, in the actual clinical operation, the application of laparoscopic surgery has many risks of complications, and the application of this operation has high requirements for medical staff and operating physicians. Therefore, in order to ensure the safety of laparoscopic surgery and reduce the trauma suffered by patients to the greatest extent, it is necessary to listen to the necessary nursing intervention for patients, strengthen the programmatic management of surgical patients, improve the quality of nursing, and promote the postoperative recovery of patients.

At present, there are many clinical nursing models, but in the management of laparoscopic surgery, there are few management models with notable effects. Among them, programmed management has the advantages of high efficiency, and it has more functions, including comprehensive, dynamic, and decision-making. Feedback and other functions have notable advantages in clinical nursing. This study found that after the completion of nursing, there were differences in the scores of nursing quality of the two sets of patients, mainly because the five scores of the research set were notably higher than those of the control set, including nursing operation, psychological support, health guidance, nursing documents, and safety management (*P* < 0.05); after nursing, there were notable differences in perioperative rehabilitation indicators between the two sets, mainly the intraoperative blood loss, anal exhaust time, first defecation time, and first self-activity, and hospital stay in the study set was notably lower compared with the control set (both *P* < 0.05); the main reason for the analysis is that the programmed nursing model must go through a series of whole processes such as evaluation, diagnosis, planning, and implementation in the development process, and it is a purposeful and planned clinical nursing activity. This nursing model can not only ensure the normal progress of nursing work, but also effectively solve the problems in nursing work, and has a good application value in helping patients recover their physical and mental health. And after one-year follow-up, the readmission rate in the control set was notably lower than that in the research set (*P* < 0.05). Because the patients in the control set lacked surgical awareness during laparoscopic surgery, they were prone to have negative emotions such as anxiety and tension during the perioperative period. Not only is it easy to trigger the body's stress response, which affects the patient's prognosis, but also easily causes the patient's concern. The use of programmed nursing management in clinical practice reduces the degree of patient cooperation and compliance with nursing measures, which increases the risk of complications and affects postoperative recovery of patients. Deep learning does not require manual design of function extractors, and it can automatically extract optimal functions and has stronger abstraction and function learning capabilities. When the sample data are large, deep learning can be used to directly obtain performance evaluation results based on hypothetical input parameters. In conclusion, speed up the evaluation. The recommended measures were formulated by the procedural nursing system for general surgery laparoscopic surgery based on deep learning, and then the procedural nursing can carry out a detailed and comprehensive preoperative evaluation of the patient, and formulate a variety of scientific and reasonable nursing plans that meet the physical and mental needs of the patient. The actual needs and support of patients can improve the postoperative recovery rate of patients. At 2 hours after operation, the VAS scores of the two sets were higher, and the difference was not statistically notable (*P* > 0.05) (both *P* < 0.05); postoperatively, the incidence of complications in the control set was 20.00%, which was notably higher than that in the study set (4.00%), and the difference was statistically notable (*P* < 0.05); the main reason for the analysis was that procedural nursing was based on evidence developed on the basis of nursing, and the most basic starting point is to optimize the perioperative nursing measures, reduce the patient's surgical stress response, and shorten the patient's recovery period. The programmed nursing mainly focuses on optimizing the perioperative nursing measures in the treatment process so that patients have no negative emotions, reduce complications, shorten the hospitalization time of patients, and allow patients to recover in a short time.

In addition, this article found that the results of *Logistic* regression model analysis showed that age >60 years, operation time >3 hours, underlying diseases, and routine nursing were the risk factors for complications of general surgery laparoscopic surgery (*P* < 0.05). Patients of old age and with underlying diseases have decreased resistance and poor autoimmunity, and are prone to infection during postoperative recovery. However, in patients with longer operation time, due to the entry and exit of the operator during the operation, the wound is exposed to the outside for a longer time, which is easy to proliferate bacteria and cause infection in the patient. In addition, the elderly patients have poor self-care ability and weak mobility, and improper nursing can lead to infection. Although some research results have been achieved in this study, the departments involved in patients are relatively weak, and there are only patients with general surgery laparoscopic surgery. Therefore, in future research, it is possible to further expand the scope of selected departments for samples to analyze the general surgery abdominal cavity based on deep learning and the realization effect of the procedural nursing system for endoscopic surgery.

## 5. Conclusion

In summary, the construction of a procedural nursing system for general surgery laparoscopic surgery based on deep learning is applied to the nursing management of general surgery laparoscopic surgery, which can improve the nursing quality of patients and VAS score, and reduce the incidence of complications of patients who are >60 years old, having operation time ≥3 hours, and with underlying diseases, and routine nursing are risk factors for complications of general surgery laparoscopic surgery. Corresponding prevention and control work should be done in the procedural nursing of general surgery laparoscopic surgery based on deep learning.

## Figures and Tables

**Figure 1:** Comparison of VAS scores at different time points. Note: “a, b, c, d” in Figure 1 indicate that the same letters indicate no difference between sets (*P* > 0.05); different letters indicate differences between sets (*P* < 0.05). “#” indicates that there is a statistical difference between the two sets during this period *P* < 0.05).

**Figure 2:** Cumulative readmission rate within 1 year after surgery.

**Table 1:** Comparison of nursing quality scores.

Set	Nursing operation	Psychological support	Health guidance	Nursing instruments	Safety management
Control set (*n* = 75)	82.19 ± 2.05	74.59 ± 2.09	85.27 ± 2.38	82.35 ± 2.36	76.35 ± 2.33
Study set (*n* = 75)	95.24 ± 2.76	90.52 ± 2.29	95.46 ± 2.75	96.27 ± 2.25	90.36 ± 2.01
*t*	−32.872	−44.497	−24.265	−36.971	−39.429
*P*	<0.001	<0.001	<0.001	<0.001	<0.001

**Table 2:** Comparison of perioperative rehabilitation indicators.

Set	Intraoperative blood loss (ml)	Anal exhaust time (d)	First defecation time (d)	First self-activity (d)	Hospitalization time (d)
Control set (*n* = 75)	76.26 ± 19.58	3.52 ± 1.19	3.37 ± 1.46	2.64 ± 1.14	6.27 ± 1.41
Study set (*n* = 75)	61.47 ± 18.29	2.16 ± 0.86	1.57 ± 0.39	1.18 ± 0.49	4.62 ± 1.24
*T*	4.780	8.838	10.315	10.190	7.610
*P*	<0.001	<0.001	<0.001	<0.001	<0.001

**Table 3:** Comparison of VAS scores at different time points after operation.

Set	2 h	12 h	24 h	*F*	*P*
Control set (*n* = 75)	7.33 ± 2.24	5.98 ± 1.73^*∗*^	4.87 ± 1.52^*∗*^^&^	19.528	<0.001
Study set (*n* = 75)	7.36 ± 2.25	4.83 ± 1.44^*∗*^	2.75 ± 1.13^*∗*^^&^	22.357	<0.001
*t*	−0.082	4.425	9.694		
*P*	0.935	<0.001	<0.001		

Note: ^*∗*^means compared with this set at 2 h after operation, and means compared with this set at 12 h after operation, *P* < 0.05.

**Table 4:** Comparison of postoperative complication rates.

Set	Lung infection	Wound infection	Urine retention	Intestinal obstruction	Total incidence
Control set (*n* = 75)	3 (4.00)	4 (5.33)	5 (6.67)	3 (4.00)	15 (20.00)
Study set (*n* = 75)	0 (0.00)	1 (1.33)	1 (1.33)	1 (1.33)	3 (4.00)
*χ*2					9.091
*P*					0.003

**Table 5:** Univariate analysis of postoperative complications.

Index	Complications occur (*n* = 18)	*χ*2	*P*
*Age*		16.318	<0.001
>60 (*n* = 35)	11 (31.43)		
≤60 (*n* = 115)	7 (6.09)		

*Gender*		0.309	0.579
Male (*n* = 91)	12 (13.19)		
Female (*n* = 59)	6 (10.19)		

*Basic illness*		12.227	0.001
Yes (*n* = 50)	12 (24.00)		
None (*n* = 100)	6 (6.00)		

*Operation time (h)*		7.955	0.005
≥3 (*n* = 70)	14 (20.00)		
<3 (*n* = 80)	4 (5.00)		

*Length of hospital stay (d)*		0.168	0.682
>7 (*n* = 60)	8 (13.33)		
≤7 (*n* = 90)	10 (11.11)		

*Incision drainage*		0.050	0.822
Yes (*n* = 62)	7 (11.29)		
None (*n* = 88)	11 (12.50)		

*Nursing method*		9.091	0.003
Usual care (*n* = 75)	15 (20.00)		
Deep learning-based programmatic nursing (*n* = 75)	3 (4.00)		

**Table 6:** Multivariate analysis assignment scale.

Factor	Assign
Dependent variable	
Complication	Happened = 1; did not happen = 2
Independent variable	
Age	>60 years = 1; ≤60 years = 2
Operation time	≥3 h = 1; <3 h = 2
Basic illness	Yes = 1; No = 2
Nursing method	Routine care = 1; deep learning-based programmed care = 2

**Table 7:** Logistic regression multivariate analysis of risk factors for postoperative complications in patients with general surgery laparoscopic surgery.

Index	Results of multivariate analysis					
	*β*	*SE*	*Wald*	*OR*	*95%CI*	*P*
Age	0.826	0.325	6.613	0.482	0.316～0.532	0.003
Operation time	0.300	0.046	40.215	0.351	0.251～0.513	0.005
Basic illness	0.232	0.093	7.501	0.261	0.087～0.559	0.002
Nursing method	0.524	0.252	11.136	0.512	0.312～0.755	0.001

## Data Availability

The simulation experiment data used to support the findings of this study are available from the corresponding author upon request.
